# Relationships between Fitness Status and Blood Biomarkers in Professional Soccer Players

**DOI:** 10.1155/2022/5135817

**Published:** 2022-04-11

**Authors:** Ana Filipa Silva, Francisco Tomás González-Fernández, Halil Ibrahim Ceylan, Rui Silva, Saeid Younesi, Yung-Sheng Chen, Georgian Badicu, Paweł Wolański, Eugenia Murawska-Ciałowicz, Filipe Manuel Clemente

**Affiliations:** ^1^Escola Superior Desporto e Lazer, Instituto Politécnico de Viana Do Castelo, Viana do castelo, Portugal; ^2^Research Center in Sports Performance, Recreation Innovation and Technology (SPRINT), Melgaço 4960-320, Portugal; ^3^The Research Centre in Sports Sciences, Health Sciences and Human Development (CIDESD), Vila Real 5001-801, Portugal; ^4^Department of Physical Education and Sport, Faculty of Education and Sport Sciences, Campus of Melilla, University of Granada, 52006 Melilla, Spain; ^5^Physical Education and Sports Teaching Department, Kazim Karabekir Faculty of Education, Ataturk University, Erzurum, Turkey; ^6^University of Coimbra, Research Unit for Sport and Physical Activity, Faculty of Sport Sciences and Physical Education, Coimbra 3004-531, Portugal; ^7^Department of Exercise and Health Sciences, University of Taipei, Taipei 11153, Taiwan; ^8^Department of Physical Education and Special Motricity, Transilvania University of Brasov, Brasov 500068, Romania; ^9^Department of Physiology, Gdansk University of Physical Education and Sport, Gdansk 80-336, Poland; ^10^Department of Physiology and Biochemistry, University School of Physical Education, Wrocław 51-612, Poland; ^11^Instituto de Telecomunicações, Delegação da Covilhã, Lisboa 1049-001, Portugal

## Abstract

**Background:**

Physical conditions are recognized to be optimal after the pre-season (PS) phase in professional sports. Given that blood measures may also reveal variations, which in turn, may present associations with fitness changes.

**Objective:**

The aim of this study is to test the changes of blood markers and physical fitness outcomes at the beginning and following the PS phase. Additionally, we aimed also to analyze the associations of training adaptations between blood markers and the physical fitness measures. *Methodology*. 25 professional male soccer players (28.1 ± 4.6 years old, 2.0 ± 7.8 kg, and 176.7 ± 4.9 cm) were assessed for hematological and biochemical parameters, and physical fitness measures in the baseline and after the phase of PS.

**Results:**

Increases in platelets were observed after the PS phase (*p* = 0.001, *η*2 = 0.39). Regarding the biochemical parameters, significant increases between PS were found for creatinine (Cre) (*p* = 0.001, *η*2 = 0.66), alkaline phosphatase (ALP) (*p* = 0.001, *η*2 = 0.79), C-Reactive Protein (CRP) (*p* = 0.001, *η*2 = 0.74), cortisol (C) (*p* = 0.001, *η*2 = 0.63), and testosterone (*T*) (*p* = 0.001, *η*2 = 0.76), whereas significant decreases were found for albumin (Alb) (*p* = 0.004, *η*2 = 0.29), and calcium corrected (Ca Corr.) (*p* = 0.002, *η*2 = 0.32). Moderate correlations were found between albumin and the 5-meter linear sprint split (*r* = –0.44 (95%CI: –0.71; –0.05)) and CRP (*r* = –0.48 (95%CI: –0.74; –0.10)). Moderate correlations were found between VAMEVAL and hemoglobin (*r* = 0.44 (95%CI: 0.05; 0.71)).

**Conclusions:**

The overall physical fitness measures improved after the PS phase. Also, significant variations (decreases/increases) were observed for the case of biomchemical and hematological outcomes. Coaches should carefully consider the adaptative changes observed in blood parameters as the changes in whole organism and metabolism after specific critical phases as the PS in professional players. Thus, optimal management of stimulus/recovery can be warranted to minimize illness and injury rate and to follow the direction and dynamics of adaptative changes.

## 1. Introduction

Understanding the biological processes inherent to the characteristics of modern professional soccer is a part of the constant evolution of periodic assessments and training monitoring systems [1]. Those facts made it possible to understand the psychophysiological and locomotor demands of modern professional soccer [2]. Soccer can be classified as an intermittent team sport, combining low-intensity actions with explosive high-intensity actions present in both training and competition [3]. Accordingly, the players are required to develop a proper physical fitness related with aerobic and anaerobic fitness, power, neuromuscular strength, change-of-direction ability, and speed at a high level, aiming to achieve the optimal performance [4].

Professional male soccer players are constantly exposed to very different external stimulus that are imposed during training to prepare them to be prepared to face the high-intensity demands of a game [5, 6]. These demands are expected to induce negative biological changes, such as an increase of cortisol levels, as a response to the external stimulus imposed [7]. Such changes can be associated to significant detriments in soccer technical skills execution and physical performance, as a consequence of accumulated fatigue [8, 9]. In fact, a recent study revealed that the participation in a single soccer match, produces detriments in physical performance due to the exposure to specific high-intensity external load measures [8]. However, different contextual factors may influence male players performance during the season and must always be considered [10].

Nevertheless, it is important to highlight that all coaches and practitioners expect to observe significant changes (in this case, improvements) to occur in players after the PS phase. Regarding this topic, soccer coaches and practitioners usually monitor and operationalize high training load (in both soccer practice and strength training), during the PS phase [11, 12]. Typically, this kind of training monitoring produces positive biological adaptations on players, allowing them to cope with the demands imposed throughout the soccer season [13].

Given the statements mentioned above, it is important to consider the implementation of periodic assessments. Thus, it allows coaches and practitioners to have a general overview of the current physical fitness status of their teams, and a detailed information regarding each athlete [14, 15]. Usually, it is preferred to conduct field tests that are capable of assessing physical fitness status. Tests such as the VAMEVAL and the 30-15 intermittent fitness, linear sprinting, and the countermovement jump (CMJ), are normally used in periodic assessments for analyzing the cardiorespiratory, speed, and power capacities of soccer players [16, 17]. On the other hand, a more invasive assessment of biological changes, such as blood biomarkers, allows to understand the individual responses to the training stimulus imposed in high-performance athletes [18].

There are different biochemical and hematological parameters that have an important role in athlete's responses to training. Indeed, some hematological measurements are regularly correlated to players' endurance capacity. For instance, the reduced aerobic performance might be partly caused by an increased Ht and Hb concentration, showing a blood hemoconcentration adaptation [19]. Those measures may assume an even important role regarding their changes during the PS phase, as the aerobic capacity is intended to positively improve [20]. As in high-performance context, the athletes are subjected to tight schedules, coaches and practitioners have to plan recovery strategies to prevent injury or illness [21]. In this case, biochemical parameters are normally used to monitor the catabolic and anabolic status of players through the analysis of cortisol and testosterone, respectively [22]. The C-Reactive protein (CRP) is an important measure to be analyzed as it is linked to acute inflammatory processes and provides useful data regarding the severity of the injury and/or trauma that caused the inflammatory status [23, 24]. The presence of basophils, neutrophils, lymphocytes, monocytes, and eosinophils constitutes a relevant role for the recovery process from injury and illness [18].

For instance, the evidences from the recent study performed on elite soccer players revealed that among other biochemical markers, the creatinine levels were significantly greater in those players experiencing greater match and training intensities [25]. Also, in the same study, no differences were found for alkaline phosphatase (ALP) [25]. Beyond that, it seems that hematological outcomes as hemoglobin, erythrocytes, and hematocrit increase during a PS phase in professional soccer contexts [26]. However, these changes do not seem to be so straightforward, as there are some studies that reported increases in hematological parameters mentioned above [26], while others reported decreases in some biochemical parameters such as total testosterone and albumin [27].

Indeed, the sports research community has conducted extensive research on the variations in different internal and external load measures, as well as on variations in physical fitness over the season [7, 28]. Furthermore, it is of great importance to consider blood biomarker variations and the potential associations of these variations with changes in physical fitness after an intense exercise program. In fact, there are several research testing dose-response relationships that measure the relationships among training intensities and physical fitness changes [7, 29, 30]. However, the overall studies on this topic, only considered subjective and objective internal intensities outcomes, such as degree of perceived exertion and heart rate measures. That is, few studies have considered the analysis of blood biomarkers in such relationships [31]. However, the abovementioned study only tested the associations between hemoglobin and training load measure, revealing that hemoglobin is a good indicator of internal load [31]. Still, to the best of our knowledge, a direct relationship between hematological and biochemical changes with physical fitness changes after a training phase is lacking.

Analyzing the blood biomarkers and physical fitness changes, as well as their interactions with physical fitness variations after the PS phase, can give new insights regarding the best strategies to manage training loads to coaches and practitioners. Considering this pertinence, our study aimed to achieve the following: (i) describe the variations of blood markers and physical fitness outcomes at the beginning and following the PS phase and (ii) describe the associations of training adaptations among blood parameters and physical fitness measures. We expected that there will be significant improvements in biochemical/hematological variables from the baseline assessment to the post-training phase and that there will be significant relationships between the outcomes of these variables and physical fitness.

## 2. Materials and Methods

### 2.1. Methodological Approach: Experimental Protocol

We have followed a within-subjects observational cohort design aiming to analyze the athletes' physical fitness and blood biomarkers variations. The study was conducted between the June and October of 2019. In the days of June 02, 2019, and September 19, 2019, baseline and after PS respectively, players were assessed considering the biological markers, hematological and biochemical parameters. Anthropometric (body weight, height, and body fat percentage (BF%), cardiorespiratory (30-15 IFT and VAMEVAL), lower-body power by use of CMJ, and sprint (20 m)) tests were performed in the baseline and after PS phase. A period of 48 h without training session/match was provided to the players in the second moment of the assessment. No trainings before occurred in the case of the beginning of the PS.

### 2.2. Participants

Participated in the study were 25 professional soccer players (28.1 ± 4.6 years old, 2.0 ± 7.8 kg, 10.3 ± 3.8% of body fat; 176.7 ± 4.9 cm), competing in a professional male Qatar club. We have tested the sample size of the present study using the formula developed by Hulley et al. [32] While, the mean and standard deviation values of similar studies reported in the literature [33–35] were included. In this formula, the standard effect size was calculated, and then the standardized effect size was inserted in the G∗Power (3.1.9.7) analysis program (one-sided, Power = 0.95, Effect size = 0.75, and *α* = 0.05). Accordingly, the minimum sample size was detected to be 21. Goalkeepers were excluded and five central defenders, five full-backs, six midfielders, five strikers, and four wingers were included. The inclusion criteria were (i) part of all repeated measures and assessments; (ii) no absence due to injuries or illnesses longer than the two weeks before the data collection; and (iii) must reported normal vision and do not declare any history of neuropsychological impairments. Participants were ensured with detailed information about the experimental design and protocol; they were informed to not take any supplementation or drugs during the phase of observation aiming to avoid interactions with changes in markers. From the initial analysis of 25 players, none was excluded from the final sample since all accomplished the inclusion criteria. This followed the guidelines of American Psychological Association (APA). Players also signed a free consent, after the agreement was provided. The research was performed taking into account the instructions for humans in the Declaration of Helsinki. At the same time, our study was confirmed by the Scientific Research Commission in Portugal (code CTC-ESDL-CE00118).

### 2.3. Measures

#### 2.3.1. Anthropometry

A body composition monitor (HD-351, Tanita, Arlington Heights, IL, USA) measured the player's body mass. The height of the participants was determined utilizing a stadiometer (Seca 217, Germany). The error of the instrument for body weight and height was approximately 0.1 kg and 0.1 cm, respectively. Also, the fat percentage (%) of players was estimated based on the skinfold thickness measurement method using a skinfold caliper (Harpenden, United Kingdom). The following sites were assessed: biceps, triceps, suprailiac, subscapular, supraspinal, thigh, abdominal, and calf. The estimated BF% was then calculated for each player, using Reilly's formula [36]. A researcher with ISAK 2 certification performed the assessments.

#### 2.3.2. Biological Markers

*(1) Hematological Parameters*. Participants were present at the laboratory for collecting blood samples, pre- and post-PS phase. For this, we took 15 ml of blood sample from the vein in each player's arm. The blood measurements took place in the morning hours (8:00–10:00 a.m, after overnight fasting). 3 ml of the total amount of blood drawn from each participant was placed in vacutainer tubes. These tubes contained ethylenediaminetetraacetic acid (EDTA). Centrifugation at 2500 rpm for 10 min was performed for the blood samples. The samples were kept at –80°C. A flow cytometer (FACSCalibur™, BD Biosciences, USA) was used for the analysis. The following hematological parameters were analyzed as follows: Hct: Hematocrit; Hb: Hemoglobin; RBC: Red blood cells; PLT: Platelets; MPLTV: Mean platelets volume; RCDW: Red cell distribution width; MCV: Mean corpuscular volume; MCHb: Mean corpuscular hemoglobin; MCHC: Mean corpuscular hemoglobin concentration; WBC: White blood cells; ANC: Absolute neutrophils count; ALC: Absolute lymphocytes count; AEC: Absolute eosinophils count; NEUT: Neutrophils; LYMP: Lymphocytes; MNC: Monocytes; EOS: Eosinophil; and BSO: Basophils

*(2) Biochemical Outcomes*. Seven milliliters (from the 15) were put into a vacutainer tube with gelose. A centrifugation at 2500 rpm for 10 min was performed for the blood samples. The plasma samples were kept at –80°C. The remaining 5 ml blood sample was stored as serum to be used in case of any problems such as hemolysis. We have used the BM-100 device to analyze biochemical markers (BioMaxima S.A., Poland). The researchers followed the manufacturer instructions to ensure the regular quality control. The following parameters were used as main outcomes: Na: Sodium; K: Potassium; Ca: Calcium; Ca Corr.: Calcium corrected; Cre: Creatinine; T: Testosterone; TC: C: Cortisol; ALP: Alkaline phosphatase; CRP: C-Reactive protein; Alb: Albumin; Ferritin; Total Cholesterol; C-HDL: High-density lipoprotein cholesterol; C-LDL: Low-density lipoprotein cholesterol; TG: Triglycerides

#### 2.3.3. Fitness Assessments

All physical measures were carried out on three different days, respecting a testing sequence that respected the order of the neuromuscular tests first and only after the tests with higher metabolic stress [17]. Given that the before and after PS assessments included anthropometric measures that were conducted on the day 1 of the testing battery. The CMJ, 20-meter sprint test, and the VAMEVAL tests were conducted on the following day. Three days after the mentioned physical tests, the 30-15 IF was then conducted to limit the fatigue effects of the previous assessments.

*(1) The Countermovement Jump Tests*. For the lower-body power assessment, the CMJ with both hands on hips and without hands on hips protocols was used [37, 38]. This test is valid and reliable for estimating explosive force in soccer [39]. The Force Decks v1.2.6109 (Vald Performance, Australia) were utilized to determine the CMJ performance. Each participant started the measurement in a standing position and was then desired to flex their knee to the depth they felt comfortable. The researchers asked them to perform the highest jump as possible while maintaining hip, knee, and ankle extension. Each participant had three trials. The best of these trials were evaluated for statistical analysis.

*(2) 20-Meter Sprint test (5, 10, 15 and 20 m Splits)*. For measuring the speed capacity of each player, the 20-m sprint test was conducted. A 20-meter straight line was delineated by two cones (Cone A: 0-meter line and Cone B: 20-meter line). Validity and reliability of the linear sprint tests were previously confirmed for adult soccer players in a recent systematic review [40]. Players were asked to start with feet split, using the preferred leg in front. Players were asked to perform the best effort possible and to not decelerate before crossing the end line. The sprinting time was measured using two photocells from Smart Speed brand (Fusion Sport, Australia). The players performed the 20 m sprint test three times with at least 3 minutes rest between each, and their performance between start and finish line was recorded in seconds. Moreover, the best scores of the players at the 5 m, 10 m, and 15 m splits were evaluated for further analysis.

*(3) VAMEVAL*. For conducting the VAMEVAL test, which is an incremental running test until reaching exhaustion, a circular 31.85 m radius setup with markers positioned at 20-meters apart from each other was ensured, as previously recommended [41]. The test was confirmed for reliability regarding the final outcome obtained [42]. All athletes were informed to maintain a running pace in accordance to the audio beep. Players were allowed to fail two times in reaching the expected position for the beep. The main outcome extracted was the total time to complete the test.

*(4) 30-15 IFT*. The 30-15IFT was executed to estimate the locomotor profile of the players, as well as estimate their heart rate maximum (HRmax). The 30-15IFT consists of performing 30-seconds of intense running interspersed by 15 s rest. During this recovery period, the players had to be within a 3-meter delineated space before the beginning of the new 30-seconds run. The test was confirmed for the high reliability level considering the main outcome (final velocity attained) [43]. The test finished in the case of the player does not sustain the effort or fail in to achieve the expected line with 3 sequential audible beeps. The HRmax (bpm) was estimated by utilizing Bluetooth HR sensors (Polar H10, Kempele, FI) positioned on the chest. The final velocity at 30-15IFT was collected for further data treatment [16].

#### 2.3.4. Statistical Procedures

The data treatment and analysis were performed in Statistica program (version 13.1, USA). The analysis of variation between baseline and after PS was conducted by one-way analysis of variance in repeated measures. Moreover, partial eta square (Fs) was used for the effect size. The magnitude of partial eta squared was classified as follows: Fs 0.00–0.02, low; Fs 0.02–0.06, intermediate; and Fs 0.06–0.14 great [44]. The correlations between outcomes (changes between baseline and following PS) were determined utilizing the Pearson correlation coefficient (*r*) [45]. The percent of variation was determined as: blood biomarkers [100 − (post *∗* 100)/pre)]; physical fitness [100 − (post *∗* 100)/pre)]. Thus, the correlations were not tested between the actual hematological and physical outcomes of the two moments, but between the percentage of change (post-pre) occurring in both type of variables. Moreover, multiple regression analysis (MLRA) was executed aiming to identify model of blood biomarkers' estimation considering the remaining physical fitness test with significant correlations.

## 3. Results

Regarding the biochemical parameters, the results were found that WBC (*p* = 0.041, *η*2 = 0.002), RBC (*p* = 0.098, *η*2 = 0.001), Hb (*p* = 0.085, *η*2 = 0.001), Ht (*p* = 0.079, *η*2 = 0.002), MCHbC (*p* = 0.097, *η*2 = 0.001), LYMP% (*p* = 0.033, *η*2 = 0.003), AEC (*p* = 0.059, *η*2 = 0.001), EOS% (*p* = 0.041, *η*2 = 0.002), ALC (*p* = 0.047, *η*2 = 0.002), MCV (*p* = 0.006, *η*2 = 0.014), MCHb (*p* = 0.012, *η*2 = 0.009), RBCDW(*p* = 0.031, *η*2 = 0.004), NEUT% (*p* = 0.018, *η*2 = 0.007), AMC (*p* = 0.006, *η*2 = 0.013), BASO% (*p* = 0.031, *η*2 = 0.004), ANC (*p* = 0.009, *η*2 = 0.011), and MNC% (*p* = 0.006, *η*2 = 0.013), did not have meaningful variations between the baseline and after phase of PS, the *F* < 1 in all cases. However, PLT (*p* = 0.001, *η*2 = 0.039) was the only measure revealing meaningful variations after the PS phase. Significant increases in PLT was observed after the phase of PS (Figures 1 and 2).

Regarding the biochemical parameters, another repeated measures ANOVAs was conducted. Significant increases between PS were found for creatinine (*p* = 0.001, *η*2 = 0.66), ALP (*p* = 0.001, *η*2 = 0.79), CRP (*p* = 0.001, *η*2 = 0.74), cortisol (*p* = 0.001, *η*2 = 0.63), and testosterone (*p* = 0.001, *η*2 = 0.76), whereas significant decreases were found for albumin (*p* = 0.004, *η*2 = 0.29) and calcium corrected (*p* = 0.002, *η*2 = 0.32). However, for sodium, TG, potassium, calcium, ferritin, TC, C-HDL, and C-LDL, no meaningful variations were detected after the PS phase (*p* > 0.05) (see Figures 3 and 4).  Figure 5 presents intra-individual variation (pre-post) for the main outcomes.

Regarding anthropometry measures, positive moderate correlations were observed among weight and PLT (*r* = 0.41, *p* = 0.042). For the linear sprint test, negative moderate correlations were observed among 5-meter sprint split and albumin (*r* = −0.44, *p* = 0.027) and CRP (*r* = −0.48; *p* = 0.013). Positive moderate correlations were found between 10-meter sprint split and Hb (*r* = 0.42, *p* = 0.032). In addition, negative moderate correlations were observed between 15-meter sprint split and albumin (*r* = −0.41, *p* = 0.041) and C-HDL (*r* = −0.43; *p* = 0.031). Finally, positive moderate correlations were found between 20-meter sprint split and MCHbC (*r* = 0.48, *p* = 0.014), and a negative moderate correlation was observed between 20-meter sprint split and LYMP (*r* = −0.44, *p* = 0.026).

In reference of VAMEVAL test, correlations were observed between VAMEVAL and Hb (*r* = 0.44, *p* = 0.025). For HRmax extracted from the VAMEVAL test, positive moderate correlations were found between MCHbC (*r* = 0.39, *p* = 0.049) and ALC (*r* = 0.47, *p* = 0.016). For CMJ with hands on hips performance, positive large correlations were found with RCDW (*r* = 0.65, *p* = 0.001) and albumin (*r* = 0.52, *p* = 0.007). Also, positive moderate correlations were found between CMJ with hands on hips and LYMP (*r* = 0.42, *p* = 0.034). On the other hand, for CMJ-free hands performance, negative large correlations were found with BASO (*r* = −0.51, *p* = 0.008). Also, positive large correlations were found with EOS (*r* = 0.52, *p* = 0.007) and CRP (*r* = 0.59, *p* = 0.002). Regarding the HRmax extracted from the 30-15 IFT test, it was revealed positive large correlations revealed potassium (*r* = 0.63, *p* = 0.001), and with albumin (*r* = 0.59, *p* = 0.002).

Table 1 shows the findings of a MLRA executed to analyze which % of change occurring in physical fitness outcomes could predict the % change of blood biomarkers.

## 4. Discussion

Our main results revealed that significant improvements were detected in body composition measurements, linear sprint (5 m, 10 m, 15 m, 20 m), VAMEVAL, 30-15 IFT, and CMJ test performance after the phase of PS. Moreover, meaningful changes in hematological and biochemical parameters were observed after the PS phase. Lastly, meaningful correlations were found between physical fitness and blood biomarkers.

Intense physical exercise, particularly during the PS phase may adversely affect the homeostatic balance in the body and may induce deterioration of the immune system, and undesirable changes in hematological/biochemical parameters. This can cause a state of overreaching and overtraining, which negatively has an impact on physical performance [46]. The evaluation of biochemical and hematological outcomes is very important in preventing the negative effects of high intense exercise during PS. It is also useful to adjust the training programs based on maintaining the health of athletes, and improving their optimal exercise performance [47]. The present study showed that the hematological parameters showed no significant differences (except PLT) throughout the PS phase. Our results revealed that PLT meaningfully augmented post-PS training program. The present results were confirmed by previous studies, that showed an augmentation in PLT following intensification of the exercise program [19, 33–35]. However, another study notified no meaningful differences in PLT after intense soccer training [26]. Similarly, Martín-García et al. [48] revealed that PLT values decreased following the PS in soccer. The same researchers also observed that decreases in PLT were accompanied by a decrease in circulating inflammation-related proteins as a result of proteomic analysis. The increase in PLT in the current research can be justified by a study conducted by Heber and Volf [49], in which they asserted that shear stress and increase in oxidative stress may trigger the increase in PLT. Exercise-activated PLT contributes to the release of growth factors and proinflammatory mediators. Moreover, increasing PLT after strenuous exercise can be associated with the development in exercise performance. This can be justified by the release of ergogenic mediators and by the stimulus for augmenting the performance improving nitric oxide into the body circulation [50]. Furthermore, our results revealed that creatinine [25] and alkaline phosphatase [25, 51, 52] increased after PS phase or intense soccer exercises. These studies are consistent with the results of our study. CRP is a very prevalent inflammatory markers associated with the acute-phase respond [53]. The present study revealed that CRP augmented after the PS phase. Compatible with the findings of the present study, the research on elite soccer players conducted by Martín-Sánchez et al. [54] showed that CRP increased after the PS phase. Contrary to our study, previous studies demonstrated that CRP concentration decreased due to the anti-inflammatory effect of exercise after prolonged intense exercise [53, 55]. On the other hand, recent studies revealed that acute intense training caused provisional increases in CRP level, and these increases were due to the cytokines, such as substantially interleukin-6 [53, 56]. It was observed that markers related to muscle damage and inflammation such as CRP and ALP augmented following PS phase. Lastly, the elevation in CRP and ALP in our research can be related to acute exercise performed 12 hours before the second blood draw (end of the PS phase). Also, cortisol and testosterone are hormonal parameters associated with psychophysiological stress. Recent studies revealed that cortisol and testosterone were frequently used in the evaluation of anabolic and catabolic balance [57–60]. The previous studies showed that the intensification of training demands in the PS phase seem to exert a significant catabolic environment, which translates to a raise of cortisol and reduction in the testosterone [61, 62]. However, our results revealed an increase in both cortisol and testosterone hormone. This result is in line with recent studies that emphasized that establishing this balance (anabolic and catabolic) during the PS is important for the quality of soccer-related physical performance throughout the season [47, 58].

The PS is an appropriate phase for improving player's body composition [63]. Recent studies showed that low body fat percentage in soccer (depending on each field position) is important for maximizing sprint [64–66], high-speed running distance [65, 67], vertical jump [68], and aerobic fitness performance in soccer players [65, 66, 69]. Our results revealed significant decreases of body composition measurements. This is affirmed by previous studies [63, 64, 70–73]. Body fat loss in soccer players in the PS was mostly related to the type and training intensity. It was recently observed that the total energy expenditure of PS explained 45% of the variance in body fat percentage. Accordingly, increased energy expenditure reflected the upregulation of aerobic metabolism through the exercise workload, which was a major mediator of substrate utilization [63]. Caldwell and Peters [64] explained that the reason for the loss in body fat after the PS can be associated with the levels aerobic and anaerobic attained in the PS phase. Moreover, the reason for fat loss may be stemmed from the characteristic structure of soccer matches, which has been reported in previous studies. The intermittent structure of soccer matches requires high demands on the aerobic energy systems (90%) that trigger high level of fat burning and accordingly, ensure the entry of free fatty acids into the bloodstream. This increases utilization of fat as energy in soccer matches may promote a reduction in body fat [51, 62, 63].

Furthermore, the current study showed that the PS phase improved the 20 m linear sprint (5 m, 10 m, 15 m, 20 m) performance. Previous studies examining changes in linear sprint performance after PS showed inconsistent results. Consistent with the present study, Caldwell and Peters [64] indicated that line sprint performance was improved after the phase of PS. A recent study [7] also revealed large improvements in 20-m sprint test after the PS training phase in elite players. In contrast, other study [72] found no significant improvement in sprint performance after PS. The augment in lower limb strength and changes in morphological structures of the body may support the improvement in linear sprint performance of soccer players [66, 74].

Our findings revealed that the VAMEVAL and 30-15 IFT tests improved significantly between assessments. There are similar studies in the literature with our results. For instance, in a study [70], an increase in maximal aerobic speed determined by VAMEVAL test was noted after the PS phase. Previous study showed that 30-15 IFT and VAMEVAL test performance moderately improved after the phase of PS [7]. Our study revealed an increase of 5.4% in the VAMEVAL test, and 6.5% in the 30-15 IFT test performance. Similarly, it was previously observed an 8.1% increase in the aerobic fitness (VO_2_max) performance after the PS phase [58]. Also, other authors, stated that VO_2_max increased significantly by 4.5% in elite soccer player after the PS phase [75]. Previous studies, which reported higher improvement than our study and the studies mentioned above, found a 27.2% increase in endurance capacity after training process in PS [66].

Our study revealed that CMJ with hands on hips, and CMJ with free hands increased significantly after the PS phase. These results were verified by recent researches that showed that CMJ performance was improved after PS [7, 58, 72, 76]. However, results are inconsistent since recent studies found no improvements in CMJ performance in team sports athletes [77–80]. In addition, it was previously shown significant decreases in CMJ performance after intensified training phase in professional [81], and amateur soccer players [82]. Recent studies suggested that the reason for the decrease in CMJ might be related to neuromuscular fatigue factors [81–83], possibly explained by training demands in the PS phase [82, 84]. The augment in CMJ in current research can be clarified by the regular application of weight training which can induce leg muscle strength improvements [64].

There are limited studies analyzing the relations between physical fitness measures and blood biomarkers. The assessment of blood biomarkers associated with oxygen transport such as Hb and MCHbC are very important for soccer performance [27]. The present study demonstrated that positive moderate correlations were found between the %change of VAMEVAL test, and the %change of hemoglobin. Also, the %change of VAMEVAL test was a predictor of the % change of hemoglobin. Hemoglobin has been tested for its relationships with aerobic fitness [57]. According to one review study, a higher hemoglobin concentration was associated with a 5% to 10% improvement in physical performance [85]. Previous studies stated that the increase in hemoglobin level was associated with better oxygen-carrying capacity of the blood, that may causes improvement in aerobic fitness performance [43, 63, 75, 77]. Additionally, Otto et al. [86] stated that maximal oxygen uptake and Hb and Hct interacted with increased sports performance, and also VO_2_max was improved increasing by about one percent for each three g/L hemoglobin augment. Our findings are not in line with some recent studies. For instance, it was recently showed that there was a negative relationship between hemoglobin level and internal loads [31]. Also, other study revealed insignificant correlations between hemoglobin levels and YYIR1 performance [46]. Saidi et al. [46] showed that the decrements of physical readiness of the elite soccer players after congested fixture can be followed by an augment in plasma volume and a decline in Hb and Ht levels. Furthermore, the % change of HRmax extracted from the VAMEVAL test was positively correlated to the % change of MCHbC and the % change of ALC. The VAMEVAL test was performed at higher heart rates after the observed phase. MCHbC indicates the hemoglobin concentration in the certain volume of RBC, and is a hematological parameter associated with hemoglobin and hematocrits. Possibly, increases in MCHbC may be justified by an augment in the hemoglobin level and a decline in the hematocrit level, resulting in a better aerobic fitness performance improvement due to greater oxygen delivery capacity [57]. The increase in hemoglobin and MCHbC following the PS phase can be explained by player's tolerance to greater training demands that are imposed during this phase [87]. Lastly, Saidi et al. [46] showed that the physical readiness may be caused by reductions in various hematological parameters, including hemoglobin levels. Therefore, after an intense training phase, the monitoring of the hemoglobin and MCHbC parameters may be extremely important for superior aerobic performance.

The current study presents some limitations. The small sample size of our study may be the first limitation. However, it was reported that the sample group consisting of professional players may be sufficient for generalizing the results [31]. Moreover, only the PS phase was examined. The blood biomarkers along with the physical performance of players can be tracked throughout the season in future studies. Regarding the effect of nutrition on blood biomarkers, no information was given about the player's nutritional status. On the other hand, the food consumption records of the players, hydration profile, and load of the matches across the phase were not determined. These should be considered as possible limitations that influence the final outcomes. Finally, some objective measures obtained in laboratory (e.g., maximal oxygen uptake, blood lactate) were not collected, thus future studies should consider these data. Despite the limitations mentioned above, no studies examined a direct relationship between physical fitness changes, and hematological/biochemical changes after an intense training phase. It is a given that longitudinal studies should be performed to analyze the associations between blood biomarkers and physical fitness parameters, taking into account the different existing player positions. Moreover, we recommend that the evaluation of hematological and biochemical markers should be controlled by moderators such as nutrition, dietary reinforcement, and rating of hydration status.

As practical implications, our results revealed that training stimulus may be associated with hematological changes which are relevant for monitoring in future occasions since some markers can be changed in regular diagnosis based on the exercise effect.

## 5. Conclusions

The PS training improved all physical fitness measures related to body composition, cardiorespiratory, speed, and power in professional soccer players. Moreover, there were no significant differences in hematological parameters after the PS phase, except for PLT, whereas significant increases/decreases in some biochemical parameters were observed after assessments. Nonetheless, meaningful correlations were observed among physical fitness changes and hematological/biochemical changes. The monitoring of physical fitness, hematological, and biochemical parameters should be performed during the PS, mainly considering the training demands occurring this phase.

## Figures and Tables

**Figure 1:** Descriptive statistics of hematological measurements (*M* ± S.D). The units of the variables are shown as follows: Hb (g/L): Ht (%): MCV (fL): MCHb (pg): MCHbC (g/dL): PLT (103/*µ*L): NEUT (%): LYMP (%): (*M*) mean, S.D.: standard-deviation. ^∗∗^*p* < 0.01.

**Figure 2:** Descriptive statistics of hematological measurements (*M* ± S.D). The units of the variables are shown as follows: WBC (10^9^/L): RBC (10^12^/L): RCDW (%): MPLTV (fL): MNC (%): EOS (%): BASO (%): ANC (10^9^/L): ALC (10^9^/L): AMC (10^9^/L): AEC (10^9^/L): M: mean, S.D.: standard-deviation.

**Figure 3:** Descriptive statistics of biochemical measures (*M* ± S.D). The units of the variables are shown as follows: Na (mmol/L): Cre (*µ*mol/L): ALP (IU/L): Alb (g/L): C (mcg/dl): T (mcg/dl): (M) mean, S.D.: standard-deviation ^∗∗^denotes significance at *p* < 0.01.

**Figure 4:** Descriptive statistics of biochemical measures (*M* ± S.D). The units of the variables are shown as follows: K (mmol/L): Ca (mmol/L): Ca Corr. (mmol/L): CRP (mcg/ml): TC (mmol/L): TG (mmol/L): C-HDL (mmol/L): C-LDL (mmol/L): ^∗^*p* < 0.05, and ^∗∗^*p* < 0.01.

**Figure 5:** Intra-individual variation for the main outcomes with significant changes. ^∗∗^*p* < 0.01.

**Table 1:** MLRA results considering the % of variation for physical measures and % of variation on the remaining blood biomarkers.

PM (% of change)	BM (% of change)	*b* ^*∗*^	SE of B^*∗*^	Adjusted *R*^2^	*F*	*p*
Body weight	PLT	0.41	0.19	13	4.66	0.04^*∗*^
5 m	MCV	−0.44	0.18	0.16	5.61	0.02^*∗*^
	CRP	−0.48	0.18	0.20	7.24	0.01^*∗*^
10 m	Hb	0.42	0.18	0.14	5.20	0.03^*∗*^
15 m	Albumin	−0.41	0.19	0.13	4.69	0.04^*∗*^
15 m	C-HDL	−0.43	0.18	0.15	5.30	0.03^*∗*^
20 m	MCHbC	0.48	0.18	0.20	7.06	0.01^*∗*^
20 m	ALC	−0.44	0.18	0.16	5.63	0.02^*∗*^
Vameval	Hb	0.44	0.18	0.16	5.73	0.02^*∗*^
HRmax	MCHbC	−0.39	0.19	0.12	4.33	0.04^*∗*^
HRmax	LYMP percentage	0.47	0.18	0.19	7.73	0.01^*∗*^
CMJ hand on hips	Hemoglobin	0.65	0.15	0.40	17.49	0.001^*∗∗*^
CMJ hand on hips	LYMP percentage	0.42	0.18	0.14	5.09	0.03^*∗*^
CMJ hand on hips	Albumin	0.52	0.17	0.24	8.76	0.006^*∗∗*^
CMJ free	EOS	0.52	0.17	0.24	8.82	0.006^*∗∗*^
CMJ free	%BASO	−0.51	0.17	0.23	8.38	0.008^*∗∗*^
CMJ free	CRP	0.59	0.16	0.30	12.32	0.001^*∗∗*^
% of change of HRmax 30-15	Potassium	0.63	0.19	0.38	16.15	0.001^*∗∗*^
% of change of HRmax 30-15	Albumin	0.59	0.16	0.32	12.42	0.001^*∗∗*^

^∗^ *p* < 0.05, ^∗∗^*p* < 0.01, PM: physical measures; BM: blood biomarkers; CMJ: 30-15 IFT: HRmax: CRP: C-HDL: Hb: PLT: MCV: MCHbC: ALC: LYMP: EOS: BASO.

## Data Availability

The raw data used to support the findings of this study may be released upon application to the Instituto Politécnico de Viana do Castelo (Portugal) (geral@esdl.ipvc.pt).
